The article "MiR-20a-5p facilitates cartilage repair in osteoarthritis via suppressing mitogen-activated protein kinase kinase kinase 2" was retracted in 2026. Reasons: concerns about the data; concerns about the results or conclusions.

# MiR-20a-5p facilitates cartilage repair in osteoarthritis via suppressing mitogen-activated protein kinase kinase kinase 2

**DOI:** 10.1080/21655979.2022.2084270

**Published:** 2022-06-15

**Authors:** Jiazhi Liu, Guo Tang, Wenjun Liu, Yi Zhou, Cunyi Fan, Wei Zhang

**Affiliations:** a Department of Orthopaedics, Shanghai Jiao Tong University Affiliated Sixth People’s Hospital, Shanghai, China; b Department of Orthopaedics, Shanghai Songjiang District Central Hospital, Shanghai, China; c Department of Orthopaedics, South Hospital of Shanghai Jiao Tong University Affiliated Sixth People’s Hospital, Shanghai, China

**Keywords:** Osteoarthritis, miR-20a-5p, Map3k2, BMSC, cartilage repair

## Abstract

Bone marrow mesenchymal stem cell (BMSC) chondrogenic differentiation contributes to the treatment of osteoarthritis (OA). Numerous studies have indicated that microRNAs (miRNAs) regulate the pathogenesis and development of multiple disorders, including OA. Nevertheless, the role of miR-20a-5p in OA remains obscure. Forty male C57BL/6 mice were divided into four groups and were surgically induced OA or underwent sham surgery in the presence or absence of miR-20a-5p. Flow cytometry was implemented to detect surface markers of BMSCs. Reverse transcription quantitative polymerase chain reaction revealed the upregulation of miR-20a-5p during BMSC chondrogenic differentiation. Western blotting displayed that miR-20a-5p inhibition decreased protein levels of cartilage matrix markers but enhanced those of catabolic and hypertrophic chondrocyte markers in BMSCs. Alcian blue staining, hematoxylin‑eosin staining and micro-CT revealed that miR-20a-5p inhibition restrained chondrogenic differentiation and miR-20a-5p overexpression promoted the repair of damaged cartilage and subchondral bone, respectively. Luciferase reporter assay identified that mitogen activated protein kinase kinase kinase 2 (Map3k2) was a target of miR-20a-5p in BMSCs. Moreover, the expression of miR-20a-5p and Map3k2 was negatively correlated in murine cartilage tissues. Knocking down Map3k2 could rescue the suppressive influence of miR-20a-5p inhibition on chondrogenic differentiation of BMSCs. In conclusion, miR-20a-5p facilitates BMSC chondrogenic differentiation and contributes to cartilage repair in OA by suppressing Map3k2.

## Highlights

- MiR-20a-5p displays a high level during chondrogenic differentiation of BMSCs.
- MiR-20a-5p inhibition suppresses chondrogenic differentiation of BMSCs.
- MiR-20a-5p overexpression facilitates cartilage repair in OA.
- MiR-20a-5p promotes chondrogenic differentiation of BMSCs by downregulating Map3k2.

## Introduction

Osteoarthritis (OA) is a joint disorder characterized by cartilage degeneration, osteophyte formation, and subchondral bone remodeling [1]. The typical symptoms caused by OA include joint pain, stiffness, swelling, and dysfunction [2]. A range of factors are considered to be responsible for the development of OA, such as aging, obesity, genetic predisposition, repeated joint trauma, and mechanical over loading [3]. The prevalence of OA is increasing, resulting in great burden on the life of many elderly individuals [4]. Drug therapies adopted for patients with OA are mainly to relieve the pain and there are no available disease-modifying treatments at present [5]. Accumulating evidence has indicated that after injury, articular cartilage has a very limited ability for self-repair and regeneration [6,7]. Hence, it is significant to find novel effective approaches for cartilage repair.

Bone marrow mesenchymal stem cells (BMSCs), an ideal source of MSCs, have been regarded as a therapeutic strategy for the repair of plentiful tissues, including the repair of damaged cartilage [8]. BMSCs are capable to differentiate into multiple cell types, including chondrocytes which participate in the formation of cartilage tissues [9]. Hence, chondrogenic differentiation of BMSCs is considered to play an indispensable role in cartilage repair [10]. Owing to the potentials of BMSCs, they are usually used in the therapy of OA. For example, BMSCs exert improved therapeutic effect on OA by activating the lysine demethylase 6A/SRY-box transcription factor 9 pathway [11]. Moreover, it was reported that regeneration of BMSCs has a significant applicant potential for treating knee OA [12].

MicroRNAs (miRNAs) are endogenous noncoding RNAs containing 18–24 nucleotides that have been reported to be potential diagnostic and therapeutic targets in the therapies of many diseases [13]. Dysregulation of miRNAs is strongly correlated with the progression of diverse physiological and pathological events [14]. Numerous studies have verified that abnormal expression of miRNAs influences the development of OA. For instance, miR-590-5p facilitates chondrocyte apoptosis, proliferation, and inflammation in OA by targeting fibroblast growth factor 18 [15]. Depletion of miR-130b promotes chondrogenic differentiation of BMSCs in OA by targeting SRY-box transcription factor 9 [16]. Recently, miR-20a-5p has been indicated to be implicated in multiple cellular processes of disorders like osteogenic and adipogenic differentiation [17,18]. Importantly, miR-20a-5p was shown to modulate tissue engineered cartilage in response to inflammatory cytokines in OA [19]. However, whether miR-20a-5p can impact BMSC chondrogenic differentiation has not been clarified and the mechanism underlying the progression of OA is unclarified.

Emerging evidence has verified that miRNAs act as crucial regulators at the posttranscriptional level by interacting with downstream messenger RNAs (mRNAs) [20]. Bioinformatics analysis displayed that mitogen-activated protein kinase kinase kinase 2 (Map3k2) is a candidate target of miR-20a-5p. Map3k2, encoding a serine/threonine protein kinase, is a critical participator in many human diseases, such as colitis [21,22]. Map3k2 was shown to mediate the activity of β-catenin in osteoblasts to promote bone formation [23]. Importantly, Map3k2 was reported to be readily detected in synovial tissue samples of patients with OA [24]. This indicated that Map3k2 might be implicated in OA pathogenesis, nevertheless, the detailed function of Map3k2 in OA is unclear.

Herein, we aimed to disclose the functions of miR-20a-5p and its mechanism in chondrogenic differentiation as well as in the repair of articular cartilage. It was hypothesized that miR-20a-5p might affect chondrogenic differentiation of BMSCs and cartilage repair by targeting certain downstream gene. Our findings might develop a novel therapeutic target for treating OA.

## Materials and methods

### Isolation, culture, and characterization of mouse BMSCs

C57BL/6 mice (male, two-week-old) were bought from Vital River (Beijing, China). All animal experiments were implemented strictly following the Guide of National Research Council for the Care and Use of Laboratory Animals and were authorized by the institutional Animal Care and Use Committee of Hubei Province Center for Disease Control and Prevention (approval number: 20221001). Isolation of BMSCs from murine femurs and tibias was conducted according to previous description [25]. Briefly, bone marrow was collected in a 15 mL centrifuge tube, washed with phosphate buffer saline and seeded at 2.5 × 10^6^ ml. Three hours later, non-adherent cells were removed using complete Dulbecco’s Modified Eagle Medium (DMEM, Corning, Corning, NY, USA). Isolated BMSCs were incubated in DMEM containing 10% fetal bovine serum (FBS, Corning) and 1% penicillin/streptomycin (Corning) at 37°C with 5% CO_2_ in a humidified incubator. To identify BMSCs, the cells were incubated at room temperature for 30 minutes with FITC-labeled antibodies against CD34, CD45, CD29, and CD44 (Abcam, Cambridge, MA, USA). Then, levels of these cell surface markers were examined by flow cytometry. A phase-contrast microscope (Nikon, Tokyo, Japan) was used for cell morphology observation.

### Alcian blue staining

A chondrogenic differentiation kit (Cyagen, Santa Clara, CA, U.S.A.) was utilized to induce chondrogenic differentiation of BMSCs. Briefly, BMSCs at the third passage were plated into 24-well plates (1 × 10^5^ cells/well) and incubated with chondrogenic medium. After incubation for 0, 7 and 14 days, BMSCs were fixed with 4% paraformaldehyde (PFA) for 15 minutes and rinsed with phosphate buffer saline followed by incubation for 40 minutes with 0.1% Alcian blue 8GX (Solarbio, Beijing, China) [26]. The optical density at 590 nm was detected.

### Cell transfection

MiR-20a-5p inhibitor and miR-NC (negative control) were obtained from GenePharma (Shanghai, China). To inhibit miR-20a-5p expression in BMSCs, 50 nM miR-20a-5p inhibitor (or miR-NC) was transfected into BMSCs. Short hairpin RNA specific to Map3k2 (Sh-Map3k2) and nonspecific control (Sh-NC) also obtained from GenePharma were transfected into BMSCs for downregulation of Map3k2. Cell transfection was conducted with Lipofectamine 2000 (Invitrogen, Carlsbad, CA, USA) [27]. Forty-eight hours post-transfection, RT-qPCR was utilized for transfection efficiency measurement.

### Reverse transcription quantitative polymerase chain reaction (RT-qPCR)

Total RNA was isolated from BMSCs and cartilage tissues using TRIzol reagent kit (Invitrogen). Reverse transcription of total RNA was achieved using Bestar^TM^ qPCR RT kit (DBI Bioscience, Shanghai, China). RT-qPCR was implemented with Fast Start Universal SYBR Green Master Mix (Roche, Shanghai, China) on a LightCycler 480 Real‐Time PCR system (Roche). Quantification of miR-20a-5p and mRNAs was performed using the 2^−ΔΔCt^ method, with U6 and GAPDH as normalization, respectively [28]. Primer sequences are listed in Table 1.

**Table 1.** Primer sequences used for RT-qPCR

Gene	Sequence (5’→3’)
mmu-miR-20a-5p forward	AGGGCTAAAGTGCTTATAGTGC
mmu-miR-20a-5p reverse	TCCTCCTCTCCTCTCCTCTC
Znfx1 forward	GCCGGGTGTCAGTTACAGG
Znfx1 reverse	CGGAAAGGAGCAGGATGGTT
Il25 forward	GGCAACTCCGTCCCACTTTA
Il25 reverse	GCAGAGTTGGCATGCACAAA
Ezh1 forward	TCAGGGTAGCTGGGCCTAAT
Ezh1 reverse	AGGGAATGGTTAGCAAGGGC
Map3k2 forward	GGAAGCTGTCCGTCACTTGA
Map3k2 reverse	GCCAGCTCTCTTCCGGTATC
Epha4 forward	AGATCCCAGCTCCCCTGAAT
Epha4 reverse	CACCAGCGATGGACAGAGTT
GAPDH forward	AGGTCGGTGTGAACGGATTTG
GAPDH reverse	GTAGACCATGTAGTTGAGGTCA
U6 forward	GTGCTCGCTTCGGCAGCACA
U6 reverse	TGGCAGGGTCCGAGGT

### Western blotting

RIPA buffer (Beyotime, Shanghai, China) was utilized for extracting total proteins from BMSCs and murine cartilage tissues. Quantification of proteins were achieved using a Bicinchoninic acid Protein Assay Kit (Beyotime). Protein samples (20 μg) were resolved with 10% sodium dodecyl sulfate polyacrylamide gel electrophoresis and transferred to polyvinylidene difluoride membranes (Invitrogen) [29]. After blocked with 5% nonfat milk, the membranes were incubated with primary antibodies against Map3k2 (ab33918, 1:10000, Abcam), Aggrecan (13880-1-AP, 1:1000, Proteintech, Chicago, USA), collagen II (Col2, ab34712, 1:1000, Abcam), collagen X (Col10, ab182563, 1:1000, Abcam), matrix metalloproteinase 13 (MMP13, ab39012, 1:3000, Abcam), ADAM metallopeptidase with thrombospondin type 1 motif 5 (ADAMTS, ab41037, 1:250) and β-actin (ab6276, 1:5000, Abcam) overnight at 4°C. After that, the membranes were incubated with corresponding horseradish peroxidase-conjugated secondary antibodies (Abcam) at room temperature for 2 hours. Eventually, protein signals were visualized using an enhanced chemiluminescence kit (Cwbiotech, Beijing, China) with an Odyssey infrared imaging system (LI-COR, Lincoln, NE, USA).

### Animal models

MiR-20a-5p or miR-NC were cloned into adeno-associated virus (AAV) vectors (HanBio, Shanghai, China). Forty C57BL/6 mice were randomly divided into four groups: Sham group + AAV-NC, Sham + AAV-miR-20a-5p, OA + AAV-NC, OA + AAV-miR-20a-5p (n = 10 mice/group). The establishment of mouse OA model was conducted as previously described [30]. In brief, after anesthesia, murine medial joint capsules were incised for implementing medial meniscus destabilization surgery. Microsurgical scissors were used to release the ligament linked to the tibial plateau, thereby inducing post-traumatic OA. Then, the joints were closed. The same procedures were conducted on mice in the sham groups without treatment for medial meniscus. After one week, AAV-NC and AAV-miR-20a-5p vectors (10 μL) were delivered intra-articularly into the knee joints, respectively. After eight weeks, mice were sacrificed via cardiac exsanguination, and murine cartilage tissues were collected.

### Hematoxylineosin (HE) staining

Murine cartilage sections were fixed with 4% PFA and embedded in paraffin. After deparaffinization and rehydration, the sections were stained with hematoxylin and eosin [31]. Observation of morphological alterations of cartilage tissues was achieved using a microscope (Nikon).

### Micro-CT

Knee joints were scanned with micro-CT (Skyscan 1176, Bruker microCT N.V., Kontich, Belgium; 4000 × 2672 pixels, 9 μm isotropic voxel size) [32]. Microtomographic data from 3-D morphometry were used to analyze the images of knee joints based on the three-dimensional parameters of trabecular bone (bone volume fraction [BV/TV, %], trabecular thickness [Tb. Th, mm] and trabecular separation [Tb. Sp, mm]).

### Luciferase reporter assay

Putative binding site of miR-20a-5p on Map3k2 was predicted by TargetScan (http://www.targetscan.org). The wild type and mutant 3’ untranslated region (3’UTR) of Map3k2 were amplified and subcloned into pmirGLO vectors (Promega, Madison, WI, USA) which were then co-transfected with miR-20a-5p inhibitor or miR-NC into BMSCs using Lipofectamine 2000 (Invitrogen). A dual luciferase® reporter assay system (Promega) was utilized for measuring the luciferase activity 48 hours post-transfection [27].

### Statistical analysis

Data are presented as the mean ± standard deviation (SD). Statistical analysis was achieved using Statistical Product and Service Solutions 21.0 software (IBM Corp., Armonk, NY, USA). Difference comparisons between two groups were analyzed by Student’s *t*-test, while those among multiple groups were examined by analysis of variance (ANOVA) followed by Tukey’s *post hoc* analysis. The expression correlation between Map3k2 and miR-20a-5p in murine cartilage tissues was identified using Pearson analysis. The value of *p* < 0.05 was considered as statistically significant.

## Results

This study aimed to investigate the functions of miR-20a-5p in BMSCs and the mouse model of OA. The potential mechanism was also under investigation. We hypothesized that miR-20a-5p might have an impact on chondrogenic differentiation of BMSCs and on cartilage damage by regulating downstream target. The results indicated that miR-20a-5p promoted chondrogenic differentiation of BMSCs and facilitated the repair of damaged cartilage by downregulating Map3k2.

### MiR-20a-5p is overexpressed during chondrogenic differentiation of BMSCs

First, flow cytometry was applied for identifying the features of BMSCs (CD34-, CD45-, CD29+, CD44+). The results indicated that the high proportion of CD44+ and CD29+ cells were considered as BMSCs (Figure 1(a)). Then, the morphology of BMSCs were observed using a microscope. It was shown that the cells had a fibroblast-like, spindle-shaped morphology and were arranged in a spiral pattern (Figure 1(b)). Chondrogenic differentiation of BMSCs was induced by chondrogenic medium and was assessed by detecting the changes in glycosaminoglycan deposition, which was a key indicator of cartilage extracellular matrix accumulation. As displayed by Alcian blue staining, glycosaminoglycan deposition was markedly enhanced with the prolonging of induction time (Figure 1(c)). In parallel, western blotting was utilized for examining protein expression of cartilage marker genes (Aggrecan and Col2). It was suggested that the protein levels of Aggrecan and Col2 were enhanced with induction time extension (Figure 1(d)). Notably, miR-20a-5p level was gradually raised along with the prolonged induction time, suggesting that miR-20a-5p is overexpressed during chondrogenic process of BMSCs (Figure 1(e)).

**Figure 1.** MiR-20a-5p is overexpressed during chondrogenic differentiation. a. Flow cytometry analysis for surface antigen expression of BMSCs. b. Morphological characteristics of BMSCs under a microscope. c. Alcian blue staining for detecting chondrogenic differentiation of BMSCs. d. Western blotting for evaluating protein levels of cartilage genes at 0, 7 and 14 days. e. RT-qPCR analysis of miR-20a-5p level. *p < 0.05, **p < 0.01.

### MiR-20a-5p inhibition suppresses chondrogenic differentiation of BMSCs

MiR-20a-5p was inhibited in BMSCs to verify whether miR-20a-5p impacts chondrogenic differentiation. MiR-20a-5p level was reduced after knockdown in cells (Figure 2(a)). After treatment with chondrogenic medium for 14 days, BMSCs were stained with Alcian blue. Notably, the staining intensity was reduced in miR-20a-5p-inhibited BMSCs (Figure 2(b,c)). Moreover, protein levels of Aggrecan and Col2 were reduced in miR-20a-5p inhibitor-transfected BMSCs compared to those in the blank control group and miR-NC-treated group, as displayed by western blotting (Figure 2(d)). Furthermore, we examined the levels of catabolic markers (ADAMTS5, MMP13) and hypertrophic chondrocyte marker (Col10) in BMSCs. As shown in Figure 2(e), protein levels of these markers were markedly enhanced in miR-20a-5p-depleted BMSCs, indicating that miR-20a-5p might suppress the formation of hypertrophic chondrocytes. Collectively, these results indicated that chondrogenic differentiation of BMSCs is suppressed after downregulating miR-20a-5p.

**Figure 2.** Depletion of miR-20a-5p inhibits chondrogenic differentiation of BMSCs. a. RT-qPCR analysis for detection of transfection efficiency of miR-20a-5p inhibitor. b-c. Alcian blue staining for assessing chondrogenic differentiation of miR-20a-5p inhibitor-transfected BMSCs. d-e. Western blotting for assessing protein levels of cartilage genes (Aggrecan and Col2), catabolic markers (ADAMTS5, MMP13) and hypertrophic chondrocyte marker (Col10) in BMSCs with above transfection. **p < 0.01, ***p < 0.001.

### Upregulation of miR-20a-5p ameliorates the condition of OA

To reveal the function of miR-20a-5p *in vivo*, establishment of a knee OA model was implemented in the C57BL/6 mice. AAV expressing miR-20a-5p or miR-NC were administrated into murine knee joints with injection. Eight weeks later, the mice were sacrificed, and knee articular cartilage tissues were collected. HE staining was carried out for histopathological observation. Relative to the normal morphology of cartilage tissues shown in the Sham group, the cartilage tissue in OA + AAV-NC group displayed a rough surface, visible cartilage fissures, and disorderly arranged chondrocytes (Figure 3(a)). Notably, in OA + AAV-miR-20a-5p group, the tissue surface became flatter, chondrocytes were elevated, and cartilage fissures were reduced (Figure 3(a)). Furthermore, as judged by modified Mankin scores, the OA model mice treated with miR-20a-5p exhibited a significant enhancement in articular cartilage thickness in comparison to OA + AAV-NC mice (Figure 3(b)). Subsequently, micro-CT was used for measuring the changes of cartilage and subchondral bone. Compared with the Sham group, the BV/TV ratio reduced and Tb. Sp enhanced in OA + AAV-NC group, while these alterations were reversed after miR-20a-5p treatment (Figure 3(c-e)), indicating that miR-20a-5p helps to repair the structure of damaged cartilage and subchondral bone in mouse OA model. This was elucidated by western blotting ulteriorly. The protein levels of cartilage marker genes (Aggrecan and Col2) were markedly reduced in OA+ AAV-NC group in comparison to those in the Sham group, and this reduction was attenuated in miR-20a-5p-treated OA mice (Figure 3(f)). In contrast, catabolic and hypertrophy markers exhibited a high level in NC-treated OA mice, whereas the high level was abated in miR-20a-5p-treated OA mice (Figure 3(g)). Collectively, miR-20a-5p might be helpful to ameliorate the formation of OA.

**Figure 3.** Upregulation of miR-20a-5p ameliorates OA. a. HE staining for histopathological observation of knee articular cartilage. b. Modified Mankin scores assigned to cartilage tissues. c-e. Micro-CT images of the mice in four groups for assessments of BV/TV, Tb. Th, and Tb. Sp. f-g. Western blotting for assessing the protein levels of cartilage markers (Aggrecan and Col2), catabolic markers (ADAMTS5, MMP13) and hypertrophic chondrocyte marker (Col10). **p < 0.01, ***p < 0.001 versus Sham + AAV-NC group; ^##^*p* < 0.01 versus Sham + AAV-miR-20a-5p group. n = 10 mice/group.

### MiR-20a-5p targets Map3k2

To reveal how miR-20a-5p exerts its impact on the progression of OA, miRDB (http://mirdb.org) was used for screening potential mRNAs containing miR-20a-5p binding site. The top five candidate mRNAs were singled out (Figure 4(a)). After that, RT-qPCR was implemented to quantify mRNA expression in miR-20a-5p-depleted BMSCs. After inhibiting miR-20a-5p in BMSCs, only Map3k2 expression was markedly upregulated (Figure 4(b)). As measured by western blotting, miR-20a-5p inhibitor raised Map3k2 protein level in BMSCs (Figure 4(c)). According to TargetScan, miR-20a-5p was elucidated to have complementary site on Map3k2 3’UTR (Figure 4(d)). The association between Map3k2 and miR-20a-5p was identified by luciferase reporter assay. It was demonstrated that after knocking down miR-20a-5p in BMSCs, the luciferase activity of Wt pmirGLO-Map3k2-3’UTR was enhanced, while that of Mut pmirGLO-Map3k2-3’UTR was not significantly influenced (Figure 4(e)).

**Figure 4.** MiR-20a-5p targets Map3k2. a. miRDB used for screening miR-20a-5p target genes. b. RT-qPCR analysis of mRNA levels of the predicted genes in miR-20a-5p-depleted BMSCs. c. Western blotting for assessing Map3k2 protein level in above cells. d. TargetScan for predicting the binding site of miR-20a-5p on Map3k2. e. Luciferase reporter assay for identifying the binding relation between Map3k2 and miR-20a-5p in BMSCs. **p < 0.01, ***p < 0.001.

### MiR-20a-5p and Map3k2 expression has a negative correlation in cartilage tissues

Subsequently, we detected levels of miR-20a-5p and Map3k2 in articular cartilage tissues by RT-qPCR. As expected, miR-20a-5p level in Sham + AAV-miR-20a-5p group was significantly higher than that in OA model groups, and compared with OA+ AAV-NC group, OA + AAV-miR-20a-5p group showed a relatively higher level of miR-20a-5p (Figure 5(a)). Conversely, Map3k2 displayed a downregulated level in Sham + AAV-miR-20a-5p group compared with Sham + AA-NC group, and its level in OA+ AAV-miR-20a-5p group was inhibited in comparison to that in OA + AAV-NC group (Figure 5(b)). In addition, Pearson analysis suggested that the expression of Map3k2 and miR-20a-5p has a negative correlation in cartilage tissues (Figure 5(c)).

**Figure 5.** The expression of Map3k2 and miR-20a-5p in murine cartilage tissues was negatively correlated. a-b. RT-qPCR of miR-20a-5p and Map3k2 levels in murine cartilage tissues. c. The expression correlation between Map3k2 and miR-20a-5p analyzed by Pearson analysis. ^&&^*p* < 0.01 versus Sham + AAV-NC group; **p < 0.01 versus Sham + AAV-NC group; ^##^*p* < 0.01 versus OA + AAV-NC group.

### Knockdown of Map3k2 rescues the miR-20a-5p inhibition-induced suppressive impacts on chondrogenic differentiation of BMSCs

Next, we explored whether miR-20a-5p facilitates chondrogenic differentiation of BMSCs by modulating Map3k2. Map3k2 protein expression was downregulated in BMSCs after transfection of Sh-Map3k2, as shown by western blotting (Figure 6(a)). Results from Alcian blue staining demonstrated that Sh-Map3k2 increased glycosaminoglycan deposition which was reduced by miR-20a-5p inhibitor (Figure 6(b,c)). Likewise, miR-20a-5p inhibitor-induced reduction in Aggrecan and Col2 protein levels in BMSCs was reversed after transfected with Sh-Map3k2 (Figure 6(d)). Additionally, knocking down Map3k2 counteracted miR-20a-5p inhibition-induced enhancement of catabolic and hypertrophy markers (Figure 6(e)). Hence, Map3k2 downregulation can reverse the suppressive influence on chondrogenic differentiation of BMSCs caused by miR-20a-5p inhibition.

**Figure 6.** Map3k2 knockdown reverses the suppressive influences of miR-20a-5p inhibition on chondrogenic differentiation. a. Western blotting of Map3k2 protein level in BMSCs transfected with Sh-Map3k2. b-c. Alcian blue staining for examining chondrogenic differentiation of BMSCs transfected with miR-NC, miR-20a-5p inhibitor or miR-20a-5p inhibitor + Sh-Map3k2. d-e. Western blotting of Aggrecan, Col2, ADAMTS5, MMP13 and Col10 protein levels in BMSCs with above transfection. **p < 0.01, ***p < 0.001 versus sh-NC/miR-NC group; ^#^*p* < 0.05, ^##^*p* < 0.01 versus miR-20a-5p inhibitor group.

## Discussion

Articular cartilage injuries may be caused by a range of factors, which lead to the formation of OA [33]. Chondrogenic differentiation of BMSCs contributes to the repair of cartilage lesions [34]. Therefore, BMSC transplantation has been considered as a promising method for treating OA [35]. Recently, miR-20a-5p attracts increasing attention and is implicated in multiple diseases [36,37]. Nevertheless, the specific role of miR-20a-5p in OA has not been reported.

In the present study, it was found that miR-20-5p displayed a high level during chondrogenic differentiation of BMSCs. Moreover, inhibition of miR-20a-5p suppressed the expression levels of Aggrecan and Col2, the components of cartilage extracellular matrix that maintain metabolic homeostasis. During the pathogenesis of OA, chondrocytes tilt toward aberrant catabolism by reducing the levels of Aggrecan and Col2 and increasing those of catabolic markers, such as MMP13 and ADAMTS5, and hypertrophic chondrocyte marker Col10, ultimately leading to articular cartilage destruction and degeneration [38]. To further elucidate the effect of miR-20a-5p on chondrogenic differentiation, we tested the expression levels of catabolic and hypertrophy markers in BMSCs. The results displayed that the expression levels of MMP13, ADAMTS5, and Col10 were markedly elevated in miR-20a-5p-depleted BMSCs. Collectively, these results indicated that miR-20a-5p might exert a protective effect on chondrocytes by promoting chondrogenic differentiation and suppressing catabolic metabolism and hypertrophic chondrocyte development. Additionally, the results from *in vivo* experiments further validated the protective role of miR-20a-5p in OA. It was shown that miR-20a-5p overexpression was favorable for the repair of damaged cartilage tissues and the maintenance of subchondral bone, confirming that miR-20a-5p upregulation restrains the pathogenesis of OA.

It is recognized that miRNAs target the 3’UTR of mRNAs by base pairing, leading to the transcriptional repression or destabilization of mRNAs [39]. To figure out the regulatory mechanism of miR-20a-5p, bioinformatics analysis was used for screening the downstream targets of miR-20a-5p. Based on a series of assays, Map3k2 was finally confirmed to be the target. Map3k2, a member of MAPK family, plays a crucial role in many disorders [22]. For example, Map3k2 and Map3k3 are inhibited by pazopanib to attenuate acute lung injuries [40]. Map3k2 is targeted by miR-335 to reduce myocardial damage, consequently helping to attenuate myocardial infarction [41]. Importantly, Map3k2 was shown to be readily detected in synovial tissue samples of patients with OA and have an impact on c-Jun N-terminal kinase signaling [24]. However, to the best of our knowledge, the detailed functions of Map3k2 and the role of miR-20a-5p/Map3k2 axis in OA have not been investigated. In this study, Map3k2 was shown to be overexpressed in murine cartilage tissues and its expression has an inverse correlation with miR-20a-5p expression. Furthermore, rescue assays demonstrated that knocking down Map3k2 could attenuate the miR-20a-5p inhibition-induced suppressive impact on chondrogenic differentiation of BMSCs. Additionally, miR-20a-5p inhibition-induced enhancement of catabolic and hypertrophic chondrocyte markers were significantly decreased in Map3k2-depleted BMSCs. These indicated that Map3k2 might suppress chondrogenic differentiation and promote hypertrophic chondrocyte development, thereby contributing to the deterioration of OA.

## Conclusion

In conclusion, we probed the functions of miR-20a-5p in chondrogenic differentiation of BMSCs as well as in the repair of damaged cartilage. MiR-20a-5p is overexpressed during BMSC chondrogenic differentiation. MiR-20a-5p depletion suppresses BMSC chondrogenic differentiation and this effect can be partially reversed by knocking down Map3k2. MiR-20a-5p overexpression is favorable for cartilage repair, thereby inhibiting the progression of OA. Our findings might develop a novel therapeutic target for OA treatment. However, in our study, it was not examined that whether there is any signaling pathway mediated by miR-20a-5p/Map3k2 axis. Additionally, more studies are needed to have a better understanding of the role of miR-20a-5p/Map3k2 axis in OA. Thus, more endeavors remain to be done in the future.

## Supplementary Material

Supplemental Material

## Data Availability

The datasets used or analyzed during the current study are available from the corresponding author on reasonable request.
